# Secure Health Monitoring Communication Systems Based on IoT and Cloud Computing for Medical Emergency Applications

**DOI:** 10.1155/2021/8016525

**Published:** 2021-12-13

**Authors:** Ali I. Siam, Mohammed Amin Almaiah, Ali Al-Zahrani, Atef Abou Elazm, Ghada M. El Banby, Walid El-Shafai, Fathi E. Abd El-Samie, Nirmeen A. El-Bahnasawy

**Affiliations:** ^1^Department of Embedded Network Systems Technology, Faculty of Artificial Intelligence, Kafrelsheikh University, Kafrelsheikh, Egypt; ^2^College of Computer Sciences and Information Technology, King Faisal University, Al-Ahsa, Saudi Arabia; ^3^Department of Electronics and Electrical Communications Engineering, Faculty of Electronic Engineering, Menoufia University, Menouf, Egypt; ^4^Department of Industrial Electronics and Control Engineering, Faculty of Electronic Engineering, Menoufia University, Menouf, Egypt; ^5^Security Engineering Laboratory, Computer Science Department, Prince Sultan University, Riyadh 11586, Saudi Arabia; ^6^Department of Computer Science and Engineering, Faculty of Electronic Engineering, Menoufia University, Menouf, Egypt

## Abstract

Smart health surveillance technology has attracted wide attention between patients and professionals or specialists to provide early detection of critical abnormal situations without the need to be in direct contact with the patient. This paper presents a secure smart monitoring portable multivital signal system based on Internet-of-Things (IoT) technology. The implemented system is designed to measure the key health parameters: heart rate (HR), blood oxygen saturation (SpO_2_), and body temperature, simultaneously. The captured physiological signals are processed and encrypted using the Advanced Encryption Standard (AES) algorithm before sending them to the cloud. An ESP8266 integrated unit is used for processing, encryption, and providing connectivity to the cloud over Wi-Fi. On the other side, trusted medical organization servers receive and decrypt the measurements and display the values on the monitoring dashboard for the authorized specialists. The proposed system measurements are compared with a number of commercial medical devices. Results demonstrate that the measurements of the proposed system are within the 95% confidence interval. Moreover, Root Mean Squared Error (RMSE), Mean Absolute Error (MAE), and Mean Relative Error (MRE) for the proposed system are calculated as 1.44, 1.12, and 0.012, respectively, for HR, 1.13, 0.92, and 0.009, respectively, for SpO_2_, and 0.13, 0.11, and 0.003, respectively, for body temperature. These results demonstrate the high accuracy and reliability of the proposed system.

## 1. Introduction

Many inventors and researchers have competed to create new systems that help specialists to diagnose and possibly treat some diseases. Diseases are usually associated with changes in some physiological parameters in the human body (e.g., heart rate, oxygen saturation, body temperature, blood pressure, etc.). The diagnosis of such diseases requires making some checks in the hospital to measure how a physiological parameter is away from the normal rates and then determine the positive or negative presence of those diseases. More deviations from normal rates are strong markers of death for a wide range of patients [1]. However, many people cannot go to the hospital continuously because they may not have enough time to go to the hospital from time to time, they have a chronic illness, or the coordinating specialist is abroad. In addition, medical care at hospitals may cost a lot. For those people, personal health devices are reliable solutions to monitor and track vital signs at home and also can call for medical help in case of emergency [2–6]. Personal health devices have an increasing interest and have become commercially available [7–9].

With recent advances in IoT and wireless sensor networks [10], many attempts have been made to deliver patient data remotely without going to the hospital [11]. This helps specialists to determine the appropriate action ahead or to send a specific equipped medical help. In emergency cases, the transmission of critical patient data can significantly impact patient life [12]. With cloud computing, which is a paradigm shift in computing and storage, IoT-based health monitoring systems found new ways of innovation [13, 14]. The cloud is the place where patient data is processed and stored, allowing vital signs of a patient to be monitored in real time or stored for historical reviews. Storing patient data in the cloud provides several benefits, including availability, reliability, and convenience at a relatively low cost [15, 16]. Various researchers [17–19] have addressed the opportunities and challenges of using cloud computing in the healthcare field. However, communication and storage of patient data within most cloud-based healthcare systems are in plain form, which puts the patient personality and privacy at stake [20]. Yi et al. [21] addressed some security threats regarding sensitive physiological data transmitted over the public channels and stored in the backend systems. Thus, an approach for delivering critical patient data to relevant healthcare providers without compromising patient privacy is needed.

The proposed system provides a secure and real-time solution for private health data records stored in the cloud. IoT biosensors are used to capture key biological parameters (heart rate, blood oxygen saturation (SpO_2_), and body temperature) from a patient at a comfortable home. Then, an IoT-based microcontroller encrypts, processes, and delivers secure health records to the public cloud. On the other side, only specialists at trusted healthcare centers can monitor the biological parameters of the patient in real time. Also, they can review historical records to predict any unusual activities and also can assign precautions to prevent any emergency cases. The proposed health monitoring system targets several patients with medical issues, such as patients in accidents or emergency places, patients with motion disabilities, patients with chronic illness, patients whose doctors are abroad, or elders who need continuous monitoring.

Securing patient data is achieved using the AES algorithm, which is a symmetric encryption algorithm that offers an excellent compromise between encryption speed and security [22]. AES algorithm is employed in the proposed system to secure patient data before storing it in the cloud. This ensures data integrity and privacy and the secure distribution of patient data in public networks.

Although there are plenty of researches and papers on the topic of health monitoring, our research, unlike most monitoring systems, adds some key contributions in the field that are as follows:

- A low cost and accurate health monitoring system is implemented to monitor the heart rate, blood oxygen saturation, and body temperature of patients without the need to be in direct contact with specialists
- Multiple medical sensors are incorporated with a compact and powerful microcontroller chip in a small-sized device with the help of IoT infrastructure. So, the implementation is simple and, at the same time, effective
- Medical measurements are encrypted before transmission to cloud storage. So, the proposed framework keeps the privacy and integrity of patient data
- End-to-end security for medical records is ensured between the patient node and the healthcare center
- The proposed system relies on a Wi-Fi-based connection, which provides fast communication between the patient module and the specialists module with low power consumption compared to other technologies

The rest of this paper is organized as follows.  Section 2 discusses some preliminaries in the context of the research work.  Section 3 gives the previous studies related to the proposed system.  Section 4 presents the proposed health monitoring system, layers, and actors of the system. System implementation is introduced in Section 5. In Section 6, the experimental results are discussed. Finally, the paper conclusion is given in Section 7.

## 2. Preliminaries

### 2.1. Blood Oxygen Saturation

Body cells and tissues need oxygen to live. Oxygen is carried from the lungs and absorbed into the Red Blood Cells (RBCs). Hemoglobin is the protein that carries oxygen in the RBCs and transports it throughout the body. The heart pumps oxygenated blood from the left ventricle to the whole body cells and tissues through the circularity system. It receives the deoxygenated blood and pumps it towards the lungs again to be oxygenated during the inhalation process. Blood oxygen saturation, termed SpO_2_, is an estimation of the amount of oxygen dissolved in the blood, which is described as the percentage of oxygenated hemoglobin to the total amount of hemoglobin, expressed as

(1) $$\begin{array}{c} {\text{SpO}}_{2}\left(\%\right)=\frac{{\text{HbO}}_{2}}{{\text{HbO}}_{2}+\text{Hb}}\times 100. \end{array}$$

SpO_2_ is one of the clinical vitals preferably measured by specialists to determine how much oxygen is saturated in the blood. Normal oxygen saturation for most healthy persons is 94% to 100% at sea level. SpO_2_ is a key indicator for the effectiveness of the respiratory system, and it can aid in the detection of hypoxemia. Furthermore, SpO_2_ level can help in the early detection of COVID-19 pneumonia [23, 24], which may cause initially unnoticeable low arterial oxygen saturation. The author in [23] reported that COVID-19 pneumonia patients have oxygen saturations as low as 50%.

The SpO_2_ level is commonly measured by a pulse oximeter, which has a Light Emitting Diode (LED) to shine the light through the fingertip and a photodetector (PD) to measure the amount of the reflected light. The structure of the pulse oximeter is depicted in Figure 1. When the light is emitted from the LED through the fingertip, some of the light is absorbed by the blood and the other amount is reflected to the PD.  Figure 2 describes the resulting waveform of the output of the PD, which has a pulsatile waveform due to the periodic change of the amount of the blood underneath the sensor due to the periodic pumping of the blood from the heart, which affects the amount of the reflected light. The more the amount of blood is, the more absorbed light and less reflected light arriving at the PD. The Direct Current (DC) component in the resulting waveform is due to the reflectance of light on bones, tissues, and other stationary parts, while the Alternating Current (AC) component represents the pulsatile change of the arterial blood that forms the photoplethysmography (PPG) signal [25–27].

With two light beams with different wavelengths, typically Red (660 nm) and Infrared (IR) (880 nm), it is reported that HbO_2_ and Hb absorb the two different wavelengths with different amounts (Figure 3). Hb has a higher absorption at 660 nm, while HbO_2_ has a higher absorption at 880 nm. This characteristic reveals that the amount of absorbed light at 660 and 880 nm can be used to estimate the amount of dissolved oxygen in the blood (SpO_2_). The two separate PPG signals determined from the Red and IR LEDs are used to find the ratio *R*, which is used to calculate the SpO_2_ level [28].

(2) $$\begin{array}{c} R=\frac{{\left(\text{AC}/\text{DC}\right)}_{\text{Red}}}{{\left(\text{AC}/\text{DC}\right)}_{\text{IR}}}. \end{array}$$

The accurate estimation of SpO_2_ is based on empirical calibration with the ratio *R* for the specific device. Equation (3) is often used in the literature to approximate the SpO_2_ value based on *R* [28].

(3) $$\begin{array}{c} {\text{SpO}}_{2}\left[\%\right]=110-25\left(R\right). \end{array}$$

Another approximation to find the value of SpO_2_ using the ratio *R* is developed by *Maxim Integrated* based on empirical calibration for their medical products and is defined as [29]:

(4) $$\begin{array}{c} {\text{SpO}}_{2}\left(\%\right)=104-17\left(R\right). \end{array}$$

In our study, the MAX30102 sensor, a product of *Maxim Integrated*, is adopted to measure the SpO_2_ level and the heart rate.

### 2.2. Heart Rate

The heart rate is denoted as the frequency at which the heart pumps blood to the arteries, and it is measured by the number of contractions of the heart per minute. The heart rate is a reflection of the physical and mental state of the body. It varies conditionally according to the body physical needs, as in the case in which the oxygen saturation level is low.

Pulse oximeters can determine the frequency of the heartbeats by calculating the time between consecutive peaks in the PPG signal using a single light source (e.g., Red LED), as shown in Figure 2. The heart rate is typically measured in beats per minute (bpm). The normal heart rate of healthy adult persons is between 60 and 100 bpm, while they are at rest.

### 2.3. AES Algorithm

Data security is an essential target in everything in our lives on all applications. Data is required to be protected from assaults and intruders. Due to the great revolution of the Internet and its applications, there is a critical need to employ security techniques to secure the transmitted information. Authorized users can transmit and receive data from a distance with communication networks. To be reliable, data needs to be safeguarded from unapproved change (integrity), hidden from unlicensed access (confidentiality), and accessible to an approved entity when required (availability). Not only should the data be trusted when it is stored in a computer, but there should also be a way to preserve its privacy when it is transmitted over a communication network.

The AES ciphering algorithm is cost-effective, and it is based on the Rijndael procedure [22], which is an iterated block ciphering process with variable key size and variable block size. The key size and block size can be autonomously 192, 128, or 256 bits. The cipher key is a rectangular array with four rows and a number of columns equal to the key size divided by 32. In addition, the intermediate resulting ciphertext describes a state and it is in the shape of a rectangular array of four rows, and a number of columns equal to the block size divided by 32. The number of rounds performed on the intermediate state is related to the key size. For key sizes of 192, 128, and 256 bits, the numbers of rounds are 10, 12, and 14, respectively. Every round comprises a fixed sequence of transformations, except the last and the first rounds.

The AES comprises a number of rounds. Any round, except the final one, involves ShiftRows, SubBytes, AddRoundKey, and MixColumns functions. In the SubBytes step, a linear substitution for every byte is performed according to Figure 4. In the final round, no MixColumns operation is executed. Every byte in the array is updated using an 8-bit S-box, which provides nonlinearity in the cipher system. The S-box is derived from the multiplicative inverse over the finite Galois Field GF (2^8^), known to have good nonlinearity characteristics. The S-box is selected to prevent fixed-point as well as opposite-fixed-point attacks.

The step of ShiftRows operates on the rows of the state. It cyclically shifts the bytes in every row. For the AES process, the first row is left unaffected. Every byte of the second row is shifted a single byte to the left. Also, the third and fourth rows are shifted by offsets of two and three bytes, respectively. For the blocks of size 192 bits or 128 bits, the shifting patterns are the same. In this manner, every column of the output state of the ShiftRows step is composed of bytes from every column of the input state. In the state of the 256-bit blocks, the first row is unaffected and the shiftings for the second, third, and fourth rows are 1 byte, 3 bytes, and 4 bytes, respectively, as demonstrated in Figure 5.

In the MixColumns step, the four bytes of every column of the state are merged with a linear invertible transformation. The MixColumns function requires four bytes as input and outputs four bytes, where every input byte involves all four output bytes. With ShiftRows, MixColumns delivers diffusion in the cipher system. Every column is treated as a polynomial over GF(2^8^) and is subsequently multiplied with a fixed polynomial *c*(*x*)=3*x*^3^+*x*^2^+*x*+2. The MixColumns step can also be considered as multiplication by a particular matrix, as demonstrated in Figure 6.

## 3. Related Studies

With recent advances in cloud computing and IoT, mobile healthcare devices were developed to provide healthcare services with more flexibility and speed at a lower cost. This helps patients receive healthcare and medical treatment anytime and helps specialists to monitor their patients in real time. From the perspective of healthcare providers, the IoT has the potential to reduce device downtime through remote provision. Besides, the IoT provides efficient scheduling of the limited resources by ensuring their best use and serves more patients [30].

In this context, several researchers have developed smart medical and healthcare surveillance and monitoring architectures. Yi et al. [21] proposed a secure health monitoring system in which private health data is encrypted using AES and split into three different servers to keep the privacy of the data even if one server is compromised. This approach defends the system against both outside and inside attacks. However, it requires more computational steps regarding generating and distributing public keys among three database servers. Ali et al. [31] implemented an IoT and Android-based health monitoring system to measure the heart rate, oxygen saturation, and body temperature of patients. Measurements are sent via Bluetooth to a mobile application and can be transmitted using Wi-Fi to the Internet. They compared the results with those of a commercially available product and reported a maximum deviation of 2%.

Mohammed et al. [32] integrated IoT and cloud computing in building an ECG mobile application, which provides the end-users with visualization for their ECG signals and logging data uploaded to the specific medical cloud. A microcontroller board was used to capture the ECG signal from a patient and send it to the mobile device in a wireless manner using Bluetooth technology. ECG data is saved as a binary file into the SD card of the mobile phone, and the user has the ability to send this file to the cloud to become available for specialist inspection.

Al-khafajiy et al. [33] proposed a Smart Healthcare Monitoring System (SW-SHMS) to monitor elderly people in their homes in real time using a mobile application. It uses a pulse sensor connected to an Arduino Uno to track the heart rate and oxygen saturation of an elder. Data from a pulse sensor is transferred to a mobile device through Bluetooth. The mobile application collects vital data from wearable sensors and sends the data to the cloud for processing and storage to become available for relevant hospitals or specialists.

Gupta et al. [34] adopted IoT and a microcontroller to monitor the vital signs of the patient. They considered only one perspective, which is the ECG signal. Raspberry Pi was used to collect data from wearable sensors and send it to a MySQL database. The authors also employed the GSM wireless network to send alert messages to healthcare centers in emergency cases. Ghosh et al. [35] implemented an IoT sensing module to measure various vital signs (ECG, body temperature, and patient position). This module is connected to a local web server via a COM connection for local monitoring and it can send measurements to cloud storage for remote monitoring.

Lloret et al. [36] presented a framework to improve the life of elders that depends on several types of communication to ease their daily affairs. They proposed Ambient Assisted Living (AAL) based wireless communication sensors, which help elders to avoid dangerous situations. Elsts et al. [37] proposed a Sensing Platform for HEalthcare in a Residential Environment (SPHERE) based on IoT technology. They presented SPHERE IoT network infrastructure for healthcare in a home environment with low power wireless network performance. Moustafa et al. [38] introduced a remote monitoring solution for developing real-time control of medical devices in eHealth applications. They presented a secure, scalable, unified, and real-time infrastructure based on sensors and IoT to remotely monitor patients. Park et al. [39] presented an emergency alert and an elderly health monitoring system that encompasses active capturing of brain and body movement signals, communication signal analysis, warning, and detection processes.

Khan et al. [40] presented a healthcare model to employ IoT technology within the field of crafty wellness care. They introduced a complete and effective healthcare monitoring framework planned based on the IoT and RFID tags. Mighali et al. [41] described a reliable and smart remote monitoring system with low cost for controlling the body motility and the position of elderly people. Tuli et al. [42] suggested a novel model named HealthFog for incorporating deep learning in edge computing devices and implementing it for automatic heart disease analysis. This model delivers healthcare as a fog service through IoT devices and proficiently manages the data of heart patients. The presented model is adaptive to a variety of operation modes of quality of service (QoS) and prediction accuracy based on user demands. Sodhro et al. [43] presented an efficient and intelligent monitoring and measurement approach for medical healthcare applications by transmitting critical patient data with good QoS through wireless networks. Alabdulatif et al. [44] discussed the main concept of a smart health IoT surveillance system in real time for cloud medium.

Table 1 summarizes the different features adopted with different healthcare-monitoring-related studies in the literature. Generally, there are few contributions in the literature on medical emergency applications adopting IoT and cloud computing technologies. Some of those introduced techniques have critical problems with medical data security and real-time communication. The traditional health monitoring systems are believed not to achieve adequate security, and they are not recommended for real-time communication. In addition, they have low robustness and require more computations in medical data processing and transmission. Hence, they increase the computational overhead. Taking into account the limitations of the state-of-the-art works, an efficient IoT and cloud-computing-based secure and real-time health monitoring communication system for medical emergency applications is the main contribution of this paper. This framework consists of IoT biosensors, an IoT-based microcontroller, an AES mechanism, and cloud storage to efficiently monitor, process, protect, store, and transmit patient medical data. Moreover, the proposed system achieves real-time communication of transmitted medical data with high quality, high robustness, and low computational complexity compared to the traditional related systems.

## 4. Proposed IoT and Cloud-Computing-Based Secure Health Monitoring System

The proposed health monitoring system aims to monitor vital data from patients or elderly people, secure it, transmit it to a public cloud database, and provide a real-time monitoring dashboard for authorized caregivers or healthcare centers at any time and anywhere. The implementation of the proposed system involves a three-layer structure of different technologies. The layers of the proposed system are the patient layer, the cloud layer, and the doctor layer. The system architecture of the proposed model with the three layers is shown in Figure 7 and described as follows.

### 4.1. Patient Layer

The patient layer consists of the patient and an IoT module. The IoT module acquires vital data from medical sensors attached to the patient body, encrypts that data, and sends ciphered data to the cloud database (i.e., second layer). The IoT module consists of a number of biomedical sensors that measure the key vital data, (heart rate, blood oxygen saturation, and body temperature), and a Wi-Fi-based microcontroller that processes this vital data, encrypts it using AES algorithm and sends it directly to the cloud database over Wi-Fi without the need to a local server or an intermediate mobile application. This procedure is performed automatically without patient interaction, making it more convenient for patients with motion disabilities and elderly people.

MAX30102 [53], shown in Figure 8(a), is a high sensitivity pulse oximeter employed to measure the heart rate and blood oxygen saturation of a patient through his fingertip. DS18B20 sensor [54], shown in Figure 8(b), is used to measure body temperature. These sensors are connected to the ESP8266 NodeMCU [55] microcontroller, which controls the whole system and provides the processing and transmission functionalities (Figure 8(c)). ESP8266 NodeMCU is an emerging IoT chip with a small-size, low-cost, self-contained Wi-Fi module, high processing speed, and capability of running self-contained applications.

The ESP8266 Crypto library [56] is adopted to provide the AES implementation for the ESP8266 module. Vital data is encrypted with a 128-bit key using Cipher Block Chaining (CBC) mode, and then encoded with Base64 format. After that, it is sent to the cloud.

AES algorithm is selected to encrypt the sensor readings, because it is simple to be implemented within the hardware using the appropriate software library, unlike other encryption algorithms, which may not be supported to be implemented in the hardware devices. In addition, it provides a good compromise between the speed of computations and the complexity.

### 4.2. Cloud Layer

The cloud layer is responsible for providing a safe place for private health data. Cloud receives sensitive data from the patient layer and stores it in a ciphered form, which makes the system more robust against not only external attacks but also internal attacks that can be initiated by the cloud service provider [57]. The cloud layer is not charged in any processing of data, but it delivers data as it is to the next layer.

Firebase [58] is employed in this work. It is a real-time cloud database, acquired by Google, and intended for IoT solutions.  Figure 9 shows a screenshot of the created real-time database on Firebase, showing encoded values for heart rate, SpO_2_, and body temperature.

### 4.3. Doctor Layer

This layer enables doctors at trusted healthcare centers to monitor and track vital data in real time. This enables doctors to predict any unusual activity and it can assign precautions to prevent any emergency case. This layer is synchronized with the cloud layer to receive updates of patient data in real time, which is in a ciphered form. A backend mechanism is used to fetch and decrypt received data and deliver it to the monitoring dashboard. First, doctors should log in via a web interface to be authenticated to prevent fraud access; and then, they are directed to the monitoring dashboard. The web interface is developed using HTML5, JavaScript, BootStrap, and ASP.NET.

## 5. System Design and Implementation

The proposed system uses the MAX30102 pulse oximeter to measure the heart rate and the blood oxygen saturation by calculating the ratio of oxygenated hemoglobin to deoxygenated hemoglobin, which is then used to calculate the percentage of oxygenated blood levels (SpO_2_), as discussed in Sections 2.1 and 2.2. For the heart rate and SpO_2_ measurements, the patient is asked to put his fingertip on the finger probe shown in Figure 10. The finger probe consists of a plastic holder with a soft contact surface, which is used to fit the fingertip on the sensor. The other end of the finger probe is connected to the device circuit board. The temperature sensor is placed under the armpit of the patient, whereas this position is recommended by specialists to measure the body temperature. Also, the other end of the sensor is connected to the specified socket in the circuit board. The block diagrams describing the procedures for measuring the heart rate, SpO2, and body temperature are shown in Figures 11 and 12. The device is powered by a 3.7 V rechargeable battery, which is a good choice for small size and long-time operation. The proposed device sends the measured medical data every five seconds, periodically. So, this is an important factor that guarantees the achievement of acceptable QoS of delivering the proposed device measurements.  Figure 13 shows the complete hardware implementation of the IoT module with relevant sensors and the microcontroller being connected. The complete system flowchart is depicted in Figure 14, indicating basic actors and their roles, whereas each actor has its own functionality to achieve the system goal, as follows.

### 5.1. Sensor Module

This module involves capturing raw physiological data from the patient's body, and sends this data to a Microcontroller Unit (MCU) for processing. This module comprises two sensor types: pulse oximeter sensor and body temperature sensor. The MAX30102 pulse oximeter sensor, shown in Figure 8(a), is involved in this study to measure the heart rate and the blood oxygen saturation. The MAX30102 is a reflective pulse oximeter that includes internal LEDs, photodetectors, optical elements, and low-noise electronics with ambient light cancellation. The communication between the MAX30102 sensor and the MCU is through the I^2^C interface. DS18B20 temperature sensor, shown in Figure 8(b), is used to sense the patient skin temperature. The DS18B20 digital thermometer provides 9-bit to 12-bit Celsius temperature measurements and communicates with the MCU through the 1-Wire interface.  Table 2 shows a summary of the technical specifications for the utilized sensors.

### 5.2. IoT Module

The IoT module is the coordinator of the whole patient layer. The process flow along this module includes the following steps:

1. Receive raw physiological data from sensors through an appropriate interface (I^2^C or 1-Wire).
2. Process the received data and convert it into numerical values (heart rate, blood oxygen saturation, and body temperature).
3. Encrypt vital signs using the AES algorithm with a 128-bit key.
4. Establish a connection to the cloud database over a Wi-Fi link.
5. Send ciphered data to cloud storage.

These tasks are accomplished using the ESP8266 NodeMCU developing kit, shown in Figure 8(c). ESP8266 is an Arduino-like board with extra beneficial features, such as 802.11 b/g/n Wi-Fi support, integrated TCP/IP protocol stack, 3.3 V operating voltage, low current consumption (10 *μ*A∼170 mA), attachable flash memory (16 MB), and high processor speed (80∼160 MHz). ESP8266 is programmed using the open-source Arduino IDE in order to accomplish its commissioned tasks.

### 5.3. Cloud

The cloud is the place where patient data is stored. Firebase cloud database server is adopted in this work to store patient data, so that the IoT module can communicate with the medical organization to allow the specialist to access and diagnose patient vital signs from anywhere at any time.

### 5.4. Hospital Local Server

This entity is responsible for receiving data from cloud storage, decrypting it with the appropriate decryption key, and then delivering it to the doctor's terminal. It also holds a SQL database comprising a table for patient information and another table for login credentials in order to control access to the system and provide authorization for users according to granted permissions.

### 5.5. Doctor Terminal

It is the last destination of patient data, where vital data of the patient is examined by a specialist to determine any health issues associated with this data and assign precautions to prevent any emergency cases. First, the specialist is asked to provide his credentials to determine his roles, after which he can proceed to the monitoring dashboard to view and interact with patient data in real time. The monitoring dashboard is updated automatically with every update in the cloud database.

## 6. Experimental Results

The proposed system provides a way to keep an eye on key biological indicators of a patient on a secure and real-time basis. With the proposed system, securing patient data is assured by encrypting the data to ensure data privacy and secure distribution of patient data in public networks. The proposed system initiates the encryption process on the IoT module, as illustrated in Figure 14, and then sends the ciphered data to the cloud. The server at the trusted healthcare center is synchronized with the cloud storage, and it is notified when the cloud storage is updated. After that, the healthcare center server fetches the new data from the cloud, which is in ciphered form. Then, the healthcare center server deciphers the data using the decryption key, which is kept secret between the system and the healthcare center. Hence, if a non-trusted user tries to sniff the outgoing data or gain access to the cloud storage, he will get ciphered data that cannot be deciphered except by using the correct decryption key. Moreover, the decryption key is unique for each module, and it is hard-coded on the microprocessor program and it cannot be inferred by an attacker.

The monitoring dashboard is shown in Figure 15. It displays the received patient data in cipher form and the decrypted values.

To evaluate the accuracy and effectiveness of the proposed health monitoring system, the measurements are compared to those of a number of commercial devices: *High Care* heart rate monitor, pulse oximeter, and a medical thermometer to measure the heart rate, SpO_2_, and the body temperature. The reference devices used in the comparison are shown in Figure 16.

The two statistical analysis tools, namely, linear correlation and Bland-Altman plot, are adopted to validate the proposed system accuracy. The measurement setup is shown in Figure 17, indicating that the proposed system values appear on the laptop screen, and the reference measurements are shown in the reference device.

A number of measurement points (50 heart rate points, 50 oxygen saturation level points, and 40 body temperature points) are taken from 20 different individuals (8 males and 12 females) of different ages (4–60 years) at different times. The data points are collected and compared against the reference measurements.

The experimental and actual measurements with error for heart rate sensor are shown in Table 3. The results reveal high agreement with the reference measurements, as shown in Figure 18, demonstrating that the proposed device is highly accurate.

Similarly, the results for the SpO_2_ and body temperature sensors are shown in Table 4, Figure 19, Table 5, and Figure 20.

Moreover, the RMSE, MAE, and MRE are computed for the proposed system as follows:

(5) $$\begin{array}{c} \text{RMSE}=\sqrt{\frac{\sum_{i=1}^{K}{\left({\text{HR}}_{ref_{i}}-{\text{HR}}_{mes_{i}}\right)}^{2}}{K}}, \end{array}$$

(6) $$\begin{array}{c} \text{MAE}=\frac{1}{K}\overset{K}{\underset{i=1}{\sum }}\left|{\text{HR}}_{ref_{i}}-{\text{HR}}_{mes_{i}}\right|, \end{array}$$

(7) $$\begin{array}{c} \text{MRE}=\frac{1}{K}\overset{K}{\underset{i=1}{\sum }}\frac{\left|{\text{HR}}_{ref_{i}}-{\text{HR}}_{mes_{i}}\right|}{{\text{HR}}_{ref_{i}}}, \end{array}$$

where HR_*ref*_ is the reference measurement from the commercial device, HR_*mes*_ is the measurement from the proposed device, and *K* is the number of measurements.

The coefficient of determination, denoted as *R*^2^, is a measure of the correlation between two variables. It ranges from 0, which indicates no correlation, to 1, which indicates a perfect match.  Table 6 summarizes the results of the proposed system for the three monitored health parameters.

In addition, Tables 7–9 compare the error rates for the proposed system against those of a number of solutions in the literature. This demonstrates the high accuracy and reliability of the proposed system against the solutions in the literature and the feasibility of applying the proposed device for clinical use.

The linear correlation analysis measures the degree of the linear relationship between two variables. The linear relationship between two variables *x* and *y* is defined as;

(8) $$\begin{array}{c} y=ax+b, \end{array}$$

where *a* and *b* are the slope and the intercept of the line, respectively.

The line of the perfect match has slope = 1 and intercept = 0, i.e.,

(9) $$\begin{array}{c} y=x. \end{array}$$

Figures 21–23 show the linear correlation plots for heart rate, SpO_2_, and body temperature results, respectively. As shown in the figures, most of the measurements are close to the line of the perfect match. The statistical analysis results indicate that the fit line for measurement points closely coincides with the line of the perfect match.

Figures 24–26 show the corresponding Bland-Altman plots of the difference between measurements versus the average for the three health parameters, respectively. The plots indicate that all difference points are within the 95% limits of agreement, where the upper 95% limit of the agreement is defined as:

(10) $$\begin{array}{c} 95{\%}_{\text{upper}}=\text{mean}+1.96\times \text{SD}, \end{array}$$

and the lower 95% limit of the agreement is defined as:

(11) $$\begin{array}{c} 95{\%}_{\text{lower}}=\text{mean}-1.96\times \text{SD}, \end{array}$$

where SD is the standard deviation for the differences.

The above results indicate that the measurements of the proposed system closely coincide with the reference measurements of the commercial products.

## 7. Conclusions and Future Works

Health monitoring systems play a crucial role in the field of health care, diagnosis and early predicting issues regarding one's health. In addition, these systems are a means of cutting medical costs regarding periodical hospital checks and doctor visits. Thus, developing a system that delivers health data from the patient place to a relative or a medical specialist became a necessity with the increasing demand.

The main outcomes of this paper are as follows:

- This paper presented a secure, low-cost, real-time, and trustable health monitoring system that provides a real-time monitoring dashboard for biological indicators within a secure environment using IoT and cloud computing.
- The proposed system adopts the AES algorithm to encrypt vital signals captured from sensors before sending them to the cloud for storage.
- An ESP8266 microcontroller is utilized to carry out the processing and encryption functions and connectivity to the cloud over Wi-Fi.
- The proposed system measurements are compared with those of a commercially available *High Care* medical device.
- The results have revealed high agreement with the reference measurements.
- The RMSE, MAE, and MRE between the reference and the measured readings are computed as 1.44, 1.12, and 0.012, respectively, for HR, 1.13, 0.92, and 0.009, respectively, for SpO_2_, and 0.13, 0.11, and 0.003, respectively, for body temperature. This indicates the high accuracy of the proposed system and its reliability to monitor the health and vital signs of patients and elders at home.

We have tried to guarantee an acceptable computational complexity for the proposed system by adopting the following approaches:

- AES algorithm is selected to encrypt the sensor data, because it is simple to be implemented within the hardware using the appropriate software library, unlike other encryption algorithms, which may not be supported to be implemented in the hardware devices. In addition, it provides a good compromise between the speed of computations and the complexity.
- Wi-Fi technology is adopted in this solution, because it is faster and more reliable.
- We rely on the cloud servers as a backend for our solution as they are characterized by their super computational power, unlimited storage, high resource utilization, and low cost.
- Messages are sent from the device every 2 seconds. Each message contains a single read. Moreover, data transmission is based on TCP. So, there is no need for a retransmission mechanism, because the packets are automatically retransmitted if the transmission fails.
- The solution has three layers: patient layer, cloud layer, and doctor layer. In real cases, where many patients are enrolled into the system, each patient will have his own IoT module to connect to the cloud server. Each patient will be located inside a different patient layer. In this case, the architecture involves multiple instances of the patient layer, while the cloud layer and the doctor layer remain as single instances. The cloud and the doctor layers are constructed with high processing and large storage capabilities to support processing of a huge amount of data that could be received from the patient layers.
- In this work, we employed the Firebase cloud server, and a real-time cloud database acquired by Google and intended for IoT solutions.

However, some limitations of the proposed solution may be encountered, which may make the device fail. The failure cases include the following:

- Loss of Internet connectivity
- Loss of the direct Wi-Fi link between the node and the local access point (e.g., wrong credentials)
- Loss or drop of the power source, such that the nodes or the sensors cannot be powered up
- Misconfiguration or utilization of the sensors in a wrong way
- Operation at exceeded limits for sensors that are defined in the datasheet

Future research directions may include further development of the proposed system to monitor more biomedical aspects such as heart activity, blood pressure, and blood glucose by integrating appropriate sensors. In addition, automated diagnosis for common diseases may be integrated with the proposed device. Moreover, a framework to process encrypted data may be developed to provide decision-making about the status of individuals, while data is encrypted.

## Figures and Tables

**Figure 1:** Pulse oximeter structure.

**Figure 2:** Reflected light waveform for a single light source.

**Figure 3:** Oxygenated and deoxygenated hemoglobin absorption graph for red and infrared wavelengths [27].

**Figure 4:** SubBytes step.

**Figure 5:** ShiftRows step.

**Figure 6:** MixColumns step.

**Figure 7:** Architecture of the proposed model.

**Figure 8:** (a) MAX30102 sensor, (b) DS18B20 sensor, and (c) ESP8266 NodeMCU WiFi Devkit.

**Figure 9:** Screenshot of the real-time cloud-based database.

**Figure 10:** Finger probe used to fit the fingertip on the MAX30102 sensor. The sensor is placed inside the plastic holder.

**Figure 11:** Heart rate and SpO_2_ monitoring block diagram.

**Figure 12:** Block diagram of body temperature monitoring.

**Figure 13:** Hardware implementation of the IoT module.

**Figure 14:** Complete system implementation flowchart.

**Figure 15:** Monitoring dashboard, indicating the ciphered and decrypted values for heart rate, SpO_2_, and body temperature readings.

**Figure 16:** Reference devices. (a) Heart rate measuring device, (b) SpO_2_ measuring device, and (c) temperature measuring device.

**Figure 17:** Reading from the proposed system versus high care reading.

**Figure 18:** Heart rate comparison.

**Figure 19:** SpO_2_ level comparison.

**Figure 20:** Body temperature comparison.

**Figure 21:** Linear relationship between measured and reference HR measurements.

**Figure 22:** Linear relationship between measured and reference SpO_2_ measurements.

**Figure 23:** Linear relationship between measured and reference body temperature measurements.

**Figure 24:** Bland–Altman plot of HR.

**Figure 25:** Bland–Altman plot of SpO_2_.

**Figure 26:** Bland–Altman plot of body temperature.

**Table 1:** Summary of different features in healthcare monitoring studies.

Feature	Type	Sample studies
Monitoring mode	Local	[31–33, 35]
	Remote	[12, 21, 34]

Transmission type	Cloud-based	[21, 31, 33, 34]
	Device-to-Device	[12, 32, 35]

Communication protocol	Wi-Fi	[31, 34]
	Bluetooth	[31–33]
	Mobile cellular network	[34]
	Zigbee	[12]

Is secured	Yes	[12, 21, 45]
	No	[32–35]

Monitored sign	Respiration	[46–50]
	Heart rate & SpO2	[31, 33]
	Body temperature	[31, 35]
	ECG	[12, 32, 34, 35]
	Blood pressure	[51, 52]
	Patient position	[35, 41]

**Table 2:** Summary of technical specifications for the utilized sensors [53, 54].

Sensor	Accuracy	Resolution	Current
MAX30102	—	18 bits	Standby: 600 *μ*A IR LED: 20 mA RED LED: 20 mA

DS18B20	±0.5°C	0.0625°C	1 mA

**Table 3:** Proposed system readings versus commercial device (High Care) readings for HR.

Reading no.	Proposed system reading	Reference reading	Error (%)
1	88	88	0.00
2	107	104	2.88
3	78	78	0.00
4	100	99	1.01
5	68	67	1.49
6	107	108	0.93
7	83	82	1.22
8	88	85	3.53
9	93	91	2.20
10	78	78	0.00
11	75	76	1.32
12	78	76	2.63
13	83	81	2.47
14	65	66	1.52
15	83	84	1.19
16	78	79	1.27
17	75	75	0.00
18	83	83	0.00
19	93	95	2.11
20	65	65	0.00
21	78	77	1.30
22	125	124	0.81
23	125	127	1.57
24	88	85	3.53
25	83	85	2.35
26	88	89	1.12
27	75	75	0.00
28	107	109	1.83
29	71	71	0.00
30	75	75	0.00
31	78	77	1.30
32	83	82	1.22
33	115	117	1.71
34	116	115	0.87
35	107	107	0.00
36	115	112	2.68
37	93	92	1.09
38	100	101	0.99
39	93	93	0.00
40	115	117	1.71
41	93	91	2.20
42	78	79	1.27
43	88	88	0.00
44	109	107	1.87
45	100	100	0.00
46	107	107	0.00
47	100	99	1.01
48	83	82	1.22
49	93	92	1.09
50	107	109	1.83

**Table 4:** Proposed system readings versus commercial device (Oximeter) readings for SpO_2_ levels.

Reading no.	Proposed system reading	Reference reading	Error (%)
1	99	98	1.02
2	98	97	1.03
3	100	98	2.04
4	99	99	0.00
5	100	99	1.01
6	97	98	1.02
7	98	99	1.01
8	99	98	1.02
9	98	98	0.00
10	99	99	0.00
11	99	99	0.00
12	99	99	0.00
13	99	100	1.00
14	100	98	2.04
15	99	100	1.00
16	99	97	2.06
17	100	99	1.01
18	99	98	1.02
19	100	99	1.01
20	99	98	1.02
21	98	97	1.03
22	100	100	0.00
23	99	99	0.00
24	100	98	2.04
25	98	99	1.01
26	99	97	2.06
27	99	100	1.00
28	98	98	0.00
29	97	99	2.02
30	98	99	1.01
31	99	98	1.02
32	98	98	0.00
33	99	97	2.06
34	100	99	1.01
35	99	98	1.02
36	98	97	1.03
37	98	100	2.00
38	98	99	1.01
39	98	98	0.00
40	99	98	1.02
41	97	98	1.02
42	100	100	0.00
43	100	99	1.01
44	97	99	2.02
45	97	97	0.00
46	98	99	1.01
47	100	99	1.01
48	99	99	0.00
49	98	97	1.03
50	99	100	1.00

**Table 5:** Proposed system readings versus commercial device (medical thermometer) readings for body temperature.

Reading no.	Proposed system reading	Reference reading	Error (%)
1	34.75	34.6	0.43
2	35.5	35.4	0.28
3	33	32.9	0.30
4	35.13	35.1	0.09
5	33.5	33.7	0.59
6	35.63	35.6	0.08
7	36.63	36.5	0.36
8	35.5	35.6	0.28
9	36.5	36.4	0.27
10	35.75	35.9	0.42
11	35.25	35.4	0.42
12	35.63	35.8	0.47
13	34.75	34.8	0.14
14	35.75	35.9	0.42
15	34.5	34.5	0.00
16	32.9	32.8	0.30
17	34.75	34.7	0.14
18	33.63	33.6	0.09
19	36	36.1	0.28
20	35.5	35.5	0.00
21	33.5	33.3	0.60
22	35.5	35.4	0.28
23	34.33	34.2	0.38
24	33.25	33.2	0.15
25	35.13	35	0.37
26	35.5	35.5	0.00
27	33.75	33.9	0.44
28	36.13	36.2	0.19
29	35.63	35.6	0.08
30	34.88	34.8	0.23
31	33.88	34.1	0.65
32	35.8	36.1	0.83
33	34.75	34.8	0.14
34	35.75	36	0.69
35	35.63	35.7	0.20
36	36.13	36.1	0.08
37	35.25	35	0.71
38	35.38	35.3	0.23
39	35.25	35.1	0.43
40	35.88	36.1	0.61

**Table 6:** Summary of the proposed system results for different health parameters.

Parameter	RMSE	MAE	MRE	*R* ^2^
HR	1.44	1.12	0.012	0.992
SpO_2_	1.13	0.92	0.009	0.074
Body temperature	0.13	0.11	0.003	0.982

**Table 7:** Comparison of HR error rates for the proposed and other solutions.

Work	RMSE	MAE	MRE (%)
[59]	2.34	2.17	2.93
[31]	3.87	3.4	4.93
Proposed	1.44	1.12	1.20

**Table 8:** Comparison of SpO_2_ error rates for the proposed and other solutions.

Work	RMSE	MAE	MRE (%)
[31]	1.41	1.2	1.24
Proposed	1.13	0.92	0.93

**Table 9:** Comparison of body temperature error rates for the proposed and other solutions.

Work	RMSE	MAE	MRE (%)
[59]	0.70	0.65	0.66
[31]	0.61	0.50	1.66
Proposed	0.13	0.11	0.31

## Data Availability

The datasets generated and analyzed during the current study are available from the corresponding author upon reasonable request.
